RETRACTED

# Influence of miRNA-30a-5p on Pulmonary Fibrosis in Mice with Streptococcus pneumoniae Infection through Regulation of Autophagy by Beclin-1

**DOI:** 10.1155/2021/9963700

**Published:** 2021-09-23

**Authors:** Hanyu Liu, Yabo Li, Yingdong Zou, Xingzong Zhang, Xiongfei Shi, Zhiping Yin, Yun Lin

**Affiliations:** Department of Laboratory, Yunnan Provincial Hospital of Traditional Chinese Medicine, Kunming, Yunnan 650021, China

## Abstract

The study is aimed at observing the influence of microribonucleic acid- (miRNA-) 30a-50p on the pulmonary fibrosis in mice with Streptococcus pneumoniae infection through the regulation of autophagy by Beclin-1. Specific pathogen-free mice were instilled with Streptococcus pneumoniae through the trachea to establish the pulmonary fibrosis model. Then, they were divided into the miRNA-30a-50p mimics group (mimics group, *n* = 10) and miRNA-30a-5p inhibitors group (inhibitors group, *n* = 10), with the control group (*n* = 10) also set. Pulmonary tissue wet weight/dry weight (W/D) was detected. The content of tumor necrosis factor-*α* (TNF-*α*), interleukin- (IL-) 6, and myeloperoxidase (MPO) was determined using enzyme-linked immunosorbent assay (ELISA). Besides, the changes in the pulmonary function index dynamic lung compliance (Cdyn), plateau pressure (Pplat), and peak airway pressure (Ppeak) were monitored, and the gene and protein expression levels were measured via quantitative PCR (qPCR) and Western blotting. The expression level of miRNA-30a-5p was substantially raised in the mimics group (*p* < 0.05), but extremely low in the inhibitors group (*p* < 0.05). The mimics group had obviously raised levels of serum aminotransferase (AST), glutamic-pyruvic transaminase (GPT), alkaline phosphatase (ALP), and pulmonary tissue W/D (*p* < 0.05). Additionally, the expression levels of TNF-*α*, IL-6, and MPO were notably elevated in the mimics group, while their expression levels showed the opposite conditions in the inhibitors group (*p* < 0.05). According to the HE staining results, the inhibitors group had arranged orderly cells, while the mimics group exhibited lung injury, pulmonary edema, severe inflammatory response, and alveolar congestion. In the inhibitors group, Cdyn was remarkably elevated, but Pplat and Ppeak declined considerably (*p* < 0.05). Besides, the inhibitors group exhibited elevated messenger RNA (mRNA) levels of Beclin-1 and LC3, lowered mRNA levels of *α*-SMA and p62, a raised protein level of Beclin-1, and a markedly decreased protein level of p62 (*p* < 0.05). Silencing miRNA-30a-5p expression can promote the expression of Beclin-1 to accelerate the occurrence of autophagy, thereby treating pulmonary fibrosis in mice with Streptococcus pneumoniae infection.

RETRACTED

## 1. Introduction

Idiopathic pulmonary fibrosis (IPF), a series of heterogeneous diffuse nonneoplastic diseases, initially occurs with the feature of alveolar epithelial cell injury and then is accompanied by excessive migration, activation, and proliferation of fibroblasts in extracellular matrix remodeling [1, 2]. IPF is characterized by inflammation and fibrosis, the most representative of which is idiopathic pulmonary failure, a progressive disease with the mean survival of 3 years. Despite in-depth research, the exact potential pathogenesis of IPF remains unclear [3]. IPF is generally considered to be a persistent damage-induced disease that is most likely to cause inflammation, and then, the expansion and proliferation of fibroblasts and deposition of extracellular matrix as well as irreversible obstructive pulmonary function decline, ultimately resulting in irreversible restrictive lung function deterioration and death [4]. It is a major breakthrough on this disease that macrolide treatment has been found to be able to prevent the progression of disease and even improve pulmonary function [5], which is, however, only applicable to the patients with increased neutrophilic granulocytes in the airway. Some experiments have also manifested that neutrophilic granulocyte-induced inflammation may play a role in the pathogenesis of IPF [6]. Although previous research focuses on parenchyma, the peripheral airway and vessels are probably involved in the pathogenesis of pulmonary fibrosis [7]. According to a study, blocking inflammation can prevent neutrophilic granulocytes from flowing into the airway, repressing pulmonary fibrosis [8].

Autophagy, a programmed death method, is strictly modulated by autophagy genes and can timely scavenge the wastes produced by cells in maintaining their own life activities, which serves as a metabolic pathway [9]. Besides, autophagy can clear harmful substances in cells, and once cells are invaded, it will make the corresponding response to keep the cells stable as a defender in organisms. Now, the research of autophagy has become a hotspot in the field of biology [10]. The mechanism of action of autophagy in physiological metabolisms in organisms has not yet been fully clarified currently, but the elucidated mechanism of action and pathway can be taken as crucial guidelines for the clinical cases of such diseases as tumor and pulmonary fibrosis. At present, the therapeutic means for pulmonary fibrosis is dominated by the antagonistic treatment for early inflammatory factors, but the efficacy is less favorable. Therefore, it is a top priority to search for ideal novel treatment strategies. The achievements in the genetic research in recent years have provided new strategies for the treatment of pulmonary fibrosis. More and more studies have demonstrated that most of human genes may be regulated by microribonucleic acids (miRNAs) [11]. miRNAs, noncoding RNAs, are involved in the specific regulation of protein coding and noncoding genes as well as multiple processes, such as cell cycle, metabolism and various immune responses [12]. A study revealed that the roles of miRNAs in the pathogenesis of different diseases are fully explored and that they play important roles in physiology and various diseases and has become crucial regulators for gene expression in many diseases, with their regulatory networks receiving extensive attention in recent years [13]. Nevertheless, the specific mechanism of the influence of miRNA-30a-50p on the pulmonary fibrosis in mice with Streptococcus pneumoniae infection through the regulation of autophagy by Beclin-1 remains less clear and needs to be delved into by researchers further.

RETRACTED

The present study is aimed at exploring the influence of miRNA-30a-50p on the pulmonary fibrosis in mice with Streptococcus pneumoniae infection through the regulation of autophagy by Beclin-1 using the classical pulmonary fibrosis animal model established in mice with Streptococcus pneumoniae infection, biochemical index detection, and quantitative reverse transcription-polymerase chain reaction (qRT-PCR) and Western blotting for determining the changes in autophagy genes and proteins. It reveals the therapeutical effect of miRNA-30a-5p on the pulmonary fibrosis in mice with Streptococcus pneumoniae infection through the regulation of autophagy by Beclin-1, providing experimental bases and theoretical references for the subsequent research and development of novel drugs.

## 2. Materials and Methods

### 2.1. Common Reagents and Consumables

Specific pathogen-free (SPF) mice (Shanghai Institutes for Biological Sciences, CSA), TRIzol reagent, DEPC-treated water, SuperScript III reverse transcriptase kit and SYBR quantitative polymerase chain reaction (qPCR) mix (ABI), radioimmunoprecipitation assay (RIPA) lysis buffer (Beyotime Biotechnology), loading buffer, protease inhibitor and bicinchoninic acid (BCA) protein concentration assay kit (Biosharp), tumor necrosis factor-*α* (TNF-*α*), interleukin- (IL-) 6 and myeloperoxidase (MPO) enzyme-linked immunosorbent assay (ELISA) kit (Nanjing Jiancheng Bioengineering Institute), glyceraldehyde-3-phosphate dehydrogenase (GAPDH) and secondary antibodies (Boster Biological Technology Co., Ltd.), primary antibodies (Santa Cruz Biotechnology, Inc.), microplate reader (Thermo Fisher Scientific), 7900HT Fast qPCR instrument (Applied Biosystems) and 2500 gel imaging system, tissue homogenizer, and electrophoresis apparatus (Bio-Rad, USA) are used.

RETRACTED

### 2.2. Establishment of Animal Model and Grouping

Twenty SPF mice were selected. The mice were fed and drank freely at a temperature of 24 ± 2°C, a humidity of 56 ± 14%, and 12 hours a day and night and were reared adaptively for 1 week. Then, a pulmonary fibrosis model was established by instilling Streptococcus pneumoniae through the trachea. Streptococcus pneumoniae bacterial solution was 0.15 mL/piece (China Institute for the Control of Pharmaceutical and Biological Products, No. 31003, 2 generations of resuscitation, colony number 3 × 10^11^/L). Two weeks after modeling, the nontissues of mice showed pulmonary fibrosis and alveolitis, and the content of hydroxyproline was significantly increased. And the expression level of *α*-smooth muscle actin and collagen in the lung tissue is obviously increased, which is regarded as a successful modeling.

In adenovirus transfection, construction of miRNA-30a-5p overexpression or silencing adenovirus vector, the related gene sequence is designed and synthesized by Shanghai Jikai Gene Company. The adenovirus mother liquor is dissolved by centrifugation and diluted with a sterile phosphate buffer into an adenovirus suspension with a titer of 5 × 10^5^ TU/*μ*L, liposome 2000 was used to transfer the expression of miRNA-30a-5p to an adenovirus vector, and the relevant adenovirus was instilled into the trachea for transfection into mice, specifically divided into the miRNA-30a-5p inhibitors group (inhibitors), miRNA-30a-5p mimics group (mimics). Another normal control group was set up, and the control group was intratracheally injected with an equal volume of normal saline under the same conditions, 10 rats in each group. The experimental protocol was approved by the experimental animal ethics committee of our hospital, and each group continued to be fed for 2 weeks, and after the end of the test period, blood and lung tissue samples were collected from mice in each group. Lung tissues were preserved in 4% paraformaldehyde for HE staining in one part and the expression of genes and proteins to be tested in a -80 freezer.

### 2.3. Evaluation of Transfection Efficiency of miRNA-30a-5p in each Group of Pulmonary Tissues

miRNA-30a-5p was transfected into mice using adenoviruses, and then, the transfection efficiency of miRNA-30a-5p in the pulmonary tissues was determined via reverse transcription- (RT-) PCR. After anesthesia via intraperitoneal injection of pentobarbital sodium, appropriate numbers of pulmonary tissues were taken carefully and smashed using the tissue homogenizer, and the expression level of miRNA-30a-5p was measured to prepare for the subsequent research of the specific molecular mechanism of action of miRNA-30a-5p in pulmonary fibrosis.

RETRACTED

### 2.4. Detection of Aspartate Aminotransferase (AST), Glutamic-Pyruvic Transaminase (GPT), Alkaline Phosphatase (ALP), and Wet Weight/Dry Weight (W/D)

At the end of trial, eyeball blood was collected routinely from mice, let stand at room temperature for 30 min, and centrifuged at 3,500× g for 10 min, and the supernatant was harvested for detection of AST, ALP, and GPT. Whether these three indexes changed was observed to further indicate the progression of pulmonary fibrosis. Subsequently, the mice were anesthetized through injection of pentobarbital sodium, and an appropriate number of pulmonary tissues were taken. The surface was dried using a piece of dry sterile ultrathin white filter paper, with such smudges as water and blood removed. After the wet pulmonary tissues were weighed using an analytical electronic balance and the experimental data were recorded in each group, the tissues were carefully placed in the drying oven at 65°C and baked until the weight stayed constant, and the dry weight was measured. The weight value in each group was recorded, and the mean was obtained to calculate the pulmonary tissue W/D.

### 2.5. Detection of Inflammatory Factors in Pulmonary Tissues

After the mice were anesthetized and sacrificed, pulmonary tissues were harvested and washed using normal saline. A total of 300 mg of pulmonary tissues were taken, broken into pieces using the homogenizer containing the tissue lysis buffer prepared, and centrifuged at 2500× g for 15 min, and the supernatant was obtained to determine the changes in the levels of MPO, IL-6, and TNF-*α*. Finally, the absorbance of these indexes in each group was measured using the microplate reader, and the standard curves were plotted to analyze the content changes according to the instructions.

### 2.6. Determination of Pulmonary Function Indexes

The pulmonary function indexes were determined in each group of mice as follows: Dynamic lung compliance (Cdyn), plateau pressure (Pplat), and peak airway pressure (Ppeak) were monitored via side-stream spirometry, and the measurement was repeated for several times to calculate the mean according to the instructions of the instrument. Finally, the data obtained were analyzed in accordance with the manufacturer's specifications.

### 2.7. HE Staining

The mice to be detected were killed by dislocation, and then, pulmonary tissues were aseptically separated and fixed in 4% paraformaldehyde at 4°C for 48 h. After being washed using running water, the tissues were dehydrated using alcohol at different concentrations, embedded in paraffin, and routinely sliced into 4-5 *μ*m thick sections. Subsequently, the sections were deparaffinized; hydrated in 95%, 90%, 80%, 75%, and 50% ethano; baked dry; and stained with hematoxylin for 20 min. After separation using hydrochloric acid and ethanol solution for 30 s, the resulting tissues were stained with eosin for 12 min, separated with 90% ethanol, and sealed. Finally, the tissues were observed under a light microscope.

RETRACTED

### 2.8. Real-Time qPCR

Total RNAs were extracted from the pulmonary tissues of mice in each group using TRIzol reagent (Invitrogen), and when the purity and concentration of the RNAs were eligible, complementary deoxyribonucleic acid strands were obtained through RT (attention should be paid to the use of isopropanol). Then, the primers were amplified in the amplification system (20 *μ*L) containing 2 *μ*L of cDNAs, 10 *μ*L of mix, 2 *μ*L of primers, and 6 *μ*L of ddH_2_O for 40 cycles. Subsequently, PCR amplification was performed under the following conditions: predenaturation at 95°C for 2 min and PCR at 94°C for 20 s, 60°C for 20 s, and 72°C for 30 s for 40 cycles. The primer sequences of the target genes and the internal reference GAPDH were designed based on the sequences from the GenBank (Table 1), and the expression levels of the target genes were measured via qRT-PCR. The expression level of mRNAs in the pulmonary tissues of mice in each group was calculated using 2^-*ΔΔ*Ct^.

### 2.9. Western Blotting

A total of 150 mg of mouse pulmonary tissues were sheared into pieces, weighed, added with RIPA lysis buffer at 100 mg/mL, and homogenized. The concentration of the total proteins extracted in the pulmonary tissues in each group of mice was determined using the BCA assay kit. Subsequently, the proteins were sampled, followed by preparation of gels, and the protein samples were loaded for electrophoresis, transferred onto a membrane, and sealed and incubated with the primary antibodies in the cassette overnight. After incubation with the secondary antibodies for 1 h, the resulting proteins were added with ELC mixture freshly prepared for color development in a darkroom. Afterwards, the protein bands were processed using software, namely, they were scanned and quantified using Odyssey scanner, and protein levels were corrected using GAPDH. Finally, Western blotting bands were quantified using Image-Pro Plus 6.0, and the expression level of each protein was calculated.

### 2.10. Statistical Analysis

The raw experimental data recorded were processed by SPSS 20.0 analysis software and subjected to multiple comparisons. The experimental results obtained were expressed as mean ± standard deviation ($\bar{\chi }\pm \text{SD}$), and *p* < 0.05 indicated statistically significant differences. GraphPad Prism 5.0 was employed to plot histograms.

RETRACTED

## 3. Experimental Results

### 3.1. Transfection of miRNA-30a-5p in Each Group of Mice

To observe the transfection efficiency of miRNA-30a-5p in each group of mice, the gene expression level of miRNA-30a-5p was measured in this study. According to the results (Figure 1), the expression level of miRNA-30a-5p was notably raised in the mimics group (*p* < 0.05), while it was obviously lowered in the inhibitors group (*p* < 0.05), suggesting that the transfection effect is obvious and can be verified by subsequent experiments.

### 3.2. Serum AST, GPT, and ALP and Pulmonary Tissue W/D

Important biochemical indicators in serum AST, GPT, ALP, etc. play an important role in pulmonary fibrosis, so we use a conventional biochemical analyzer to detect their content. The results are shown in Table 2. Compared with the control group, the content of AST, GPT, ALP, and lung tissue W/D in the mimics group increased significantly (*p* < 0.05). Compared with the mimics group, the inhibitors group AST, GPT, ALP, and lung tissue W/D content significantly decreased (*p* < 0.05).

### 3.3. Inflammatory Factors in Each Group

In this study, the levels of inflammatory factors such as TNF-*α*, IL-6, and MPO were detected as shown in Table 3. Compared with the control group, the levels of the three in the mimics group were significantly increased (*p* < 0.05), and compared with the mimics group, the levels of the three in the inhibitors group were significantly lower (*p* < 0.05). It shows that lung tissue inflammatory factors are produced in large quantities in pulmonary fibrosis mice, and miRNA-30a-5p inhibitors can inhibit the production of lung tissue inflammatory factors.

### 3.4. Pulmonary Function Indexes

As shown in Table 4, compared with the control group, Cdyn in the mimics group was significantly reduced, and Pplat and Ppeak were significantly increased (*p* < 0.05). Compared with the mimics group, Cdyn in the inhibitors group was significantly increased, while Pplat and Ppeak were significantly decreased (*p* < 0.05).

### 3.5. Changes in Pulmonary Tissues Observed via He Staining

The mice in the mimics group had lung injury, pulmonary edema, severe inflammatory response, alveolar congestion, and cell injury (Figure 2(a)), while those in the inhibitors group had cells with basically normal morphology and relatively normal histological structure, without obvious pathological changes compared with the control group (Figure 2(b)).

RETRACTED

### 3.6. Gene Expression Levels of *α*-SMA, Beclin-1, LC3, and p62 Determined via RT-PCR

Using RT-PCR technology to detect changes in gene expression levels, the results are shown in Figure 3. Compared with the control group, the expression levels of LC3 and Beclin-1 genes in the mimics group were significantly reduced, and the expression levels of p62 and *α*-SMA genes were significantly increased (*p* < 0.05). Compared with the mimics group, the expression levels of LC3 and Beclin-1 genes in the inhibitors group were significantly increased (*p* < 0.05), and the expression levels of p62 and *α*-SMA genes were significantly decreased (*p* < 0.05).

### 3.7. Expressions of Autophagy-Associated Proteins

We detected the expression levels of two important autophagy proteins, and the results are shown in Figure 4. Compared with the control group, the LC3 and Beclin-1 proteins in the Mimics group were significantly reduced (p <0.05). Compared with the mimics group, LC3 and Beclin-1 proteins in the inhibitors group increased significantly (*p* < 0.05).

## 4. Discussion

Pulmonary fibrosis is a disease in the lung, which has high morbidity and mortality rates in many children and adults and the features of filling of inflammatory cells, recruitment of fibroblasts, and fibrosis can be secondary to acute lung injury such as acute respiratory distress syndrome and chronic inflammation like cystic fibrosis [14, 15]. The pathological features of pulmonary fibrosis, a fatal disease, may depend on the potential disease process, but its etiology is unclear, so that little has been known about the molecular pathway and cellular mechanism, and there are no efficacious medications or medications have significant side effects [16]. Therefore, there is an urgent need of an efficacious treatment strategy. This study explored the influence of miRNA-30a-5p on the pulmonary fibrosis in mice with Streptococcus pneumoniae infection through the regulation of autophagy by Beclin-1. miRNA-30a-5p was first transfected into mice using adenoviruses, and then the gene expression level of miRNA-30a-5p was measured to observe the transfection efficiency of miRNA-30a-5p in each group of mice. It was found that the expression level of miRNA-30a-5p was notably raised in the mimics group, while it was obviously lowered in the inhibitors group, suggesting that the transfection effect is obvious and can be verified by subsequent experiments. Since sera AST, GPT, and ALP are important indexes in pulmonary fibrosis, their content was determined using a routine biochemical analyzer in this study. According to the detection results, the inhibitors group had substantially lowered content of AST, GPT, and ALP and pulmonary tissue W/D, while they were notably elevated in the mimics group. Additionally, the levels of IL-6, TNF-*α*, and other inflammatory activation factors are associated with the development of pulmonary fibrosis. Research showed that the increase in B lymphocytes in the lung probably produces such inflammatory factors as IL-6, thus inducing pulmonary fibrosis [17]. In the present research, the levels of the inflammatory factors TNF-*α*, IL-6, and MPO were determined, and it was found that the levels of these three factors in the mimics group were obviously higher than those in the other two groups, while their levels declined distinctly in the inhibitors group, illustrating that there are massive inflammatory factors in the pulmonary tissues of pulmonary fibrosis mice and that miRNA-30a-5p inhibitors can repress the production of inflammatory factors in pulmonary factors. According to the HE staining results, the mice in the mimics group had lung injury, pulmonary edema, severe inflammatory response, alveolar congestion, and cell injury, while those in the inhibitors group had cells with basically normal morphology and relatively normal histological structure, without obvious pathological changes compared with the control group. Moreover, Cdyn was considerably elevated, but Pplat and Ppeak were notably lowered in the inhibitors group, while they showed the opposite trends in the mimics group, which are consistent with the results of the previous studies. [18]

As an evolutionarily conservative mechanism, autophagy maintains the stability of cells through eliminating misfolded/mutated or aggregated proteins and damaged organelles and it allows cells to survive under stress conditions, such as nutrition deficiency, energy deficiency, viral infection, and hypoxia [19]. There is growing evidence that autophagy is likely to help resist cancers, aging, neurodegenerative diseases, and infection [20]. miRNAs have been increasingly proven to be able to regulate cell proliferation, apoptosis, and other basic biological processes and play a pivotal role in the regulation of cell autophagy [21]. Autophagy is modulated by autophagy-associated genes and proteins, including Beclin-1, LC3, and p62, that are involved in autophagosome formation. Research proposed that positively regulating the expression of Beclin-1 gene can accelerate the occurrence of autophagy [22]. LC3, synthesized by ubiquitin-like proteins in cells, is catalyzed by Atg4 homologues to expose some amino acid residues and dissolve in the whole cell cytoplasm [23]. According to the findings in a study, a great increase in the content of p62 gene is detected in the autophagy-defective test, further revealing that the content of p62 is negatively correlated with autophagy intensity [24]. In this study, the influence of miRNA-30a-5p on the pulmonary fibrosis in mice through the regulation of autophagy by Beclin-1 was observed, and according to the gene detection results, the inhibitors group had substantially raised gene expression levels of LC3 and Beclin-1, but notably lowered gene expression levels of p62 and *α*-SMA, while the mimics group exhibited the opposite conditions. The expression levels of LC3 and Beclin-1, two important autophagy-associated proteins, were also measured in this study, and it was found that the inhibitors group had obviously elevated levels of LC3 and Beclin-1 proteins, but their levels were evidently raised in the mimics group, which is in accordance with the results of the previous studies [25]. The present study proved through a train of animal experiments that silencing miRNA-30a-5p can regulate Beclin-1 to spur the occurrence of autophagy and inhibit the production of inflammatory factors, playing a therapeutical role in pulmonary fibrosis mice.

RETRACTED

In conclusion, silencing miRNA-30a-5p may protect against pulmonary fibrosis, alleviate inflammatory cell infiltration, enhance pulmonary and biochemical functions and prevent the further progression of inflammation, and ultimately affect the progression of pulmonary fibrosis through activating Beclin-1 to regulate autophagy, so the present research provides a novel theoretical basis of prevention and treatment of pulmonary fibrosis.

## Figures and Tables

**Figure 1:** Transfection efficiency of miRNA-30a-5p. The expression level of miRNA-30a-5p is remarkably raised in the mimics group (*p* < 0.05), while it evidently declines in the inhibitors group (*p* < 0.05). ^∗^*p* < 0.05 vs. the control group, ^#^*p* < 0.05 vs. the mimics group.

**Figure 2:** HE staining results. The mice in the mimics group have lung injury, pulmonary edema, severe inflammatory response, alveolar congestion, and cell injury ((a) ×100), while those in the inhibitors group have cells with basically normal morphology and relatively normal histological structure, without obvious pathological changes compared with the control group ((b) ×100).

**Figure 3:** Gene expression levels. The inhibitors group has remarkably raised gene expression levels of LC3 and Beclin-1 (*p* < 0.05) and markedly decreased gene expression levels of *α*-SMA and p62 (*p* < 0.05), while the gene expression trends are the opposite in the mimics group. ^∗^*p* < 0.05 vs. the control group, ^#^*p* < 0.05 vs. the mimics group.

**Figure 4:** Expressions of autophagy-associated proteins. (a) Western blot result. (b) Quantification analysis of Western blot result. The expression levels of LC3 and Beclin-1 proteins are evidently raised in the inhibitors group (*p* < 0.05), but they show the opposite conditions in the mimics group. ^∗^*p* < 0.05 vs. the control group, ^#^*p* < 0.05 vs. the mimics group.

RETRACTED

**Table 1:** PCR primers.

Target gene	Primer sequence
GAPDH	F: 5′-CAGTGCCAGCCTCGTCTCAT-3′ R: 5′- AGGGCCATCCACAGTCTTC-3′
*α*-Smooth muscle actin (*α*-SMA)	F: 5′-GTCCCAGACATCAGGGAGTAA-3′ R: 5′-TCGGATACTTCAGCGTCAGGA-3′
Beclin-1	F: 5′-AATCTAAGGAGTTGCCGTTATAC-3′ R: 5′-CCAGTGTCTTCAATCTTGCC-3′
LC3	F: 5′-ACATGAGCGAGTTGGTCAAG-3′ R: 5′-GTTCATAGATGTCAGCGATG-3′
p62	F: 5′-GTGTCTTGGCATTCTTGTAG-3′ R: 5′-AGCAGAGGAAGCTCAGCTCA-3′
miRNA-30a-5p	F: 5′-TGTAAACATCCTCGACTGGAAG-3′ R: 5′-ACATTTGTAGGAGCTGACCTTC-3′

**Table 2:** Changes in AST, GPT, ALP, and W/D.

Group	AST (U/L)	W/D	ALP (U/L)	GPT (U/L)
Control	153.2 ± 6.3	3.6 ± 0.2	89.8 ± 5.2	42.3 ± 5.6
Mimics	296.8 ± 2.8^∗^	10.2 ± 1.3^∗^	205.5 ± 4.4^∗^	127.1 ± 5.7^∗^
Inhibitors	183.6 ± 3.5^#^	5.3 ± 1.9^#^	101.1 ± 5.8^#^	50.7 ± 4.5^#^

Note: the content of AST, GPT, and ALP and pulmonary tissue W/D decline markedly in the inhibitors group, while they are notably elevated in the mimics group (*p* < 0.05). ^∗^*p* < 0.05 vs. the control group, ^#^*p* < 0.05 vs. the mimics group.

**Table 3:** Levels of inflammatory factors.

Group	TNF-*α* (fmol/mL)	IL-6 (mg/L)	MPO (U/mg)
Control	33.7 ± 3.1	65.1 ± 4.1	3.5 ± 1.0
Mimics	95.9 ± 6.7^∗^	134.7 ± 5.2^∗^	14.6 ± 1.1^∗^
Inhibitors	42.0 ± 5.8^#^	75.1 ± 4.0^#^	4.6 ± 1.8^#^

Note: the levels of IL-6, TNF-*α*, and MPO are evidently elevated in the mimics group, but their levels are obviously lowered in the inhibitors group. ^∗^*p* < 0.05 vs. the control group, ^#^*p* < 0.05 vs. the mimics group.

**Table 4:** Pulmonary function indexes.

Group	Cdyn (mL/cmH_2_O)	Ppeak (cmH_2_O)	Pplat (cmH_2_O)
Control	50.7 ± 2.0	9.1 ± 1.1	8.8 ± 2.5
Mimics	24.1 ± 2.3^∗^	32.1 ± 2.2^∗^	35.1 ± 2.0^∗^
Inhibitors	46.1 ± 2.7^#^	12.5 ± 1.0^#^	15.4 ± 2.2^#^

Note: Cdyn is considerably elevated, but Pplat and Ppeak are notably lowered in the inhibitors group (*p* < 0.05), while they show the opposite trends in the mimics group (*p* < 0.05). ^∗^*p* < 0.05 vs. the control group, ^#^*p* < 0.05 vs. the mimics group.

## Data Availability

The datasets used and/or analyzed during the current study are available from the corresponding author on reasonable request.
